# Evaluation of Heavy Metals in Soil Wastewater Stream

**DOI:** 10.1155/2022/2522840

**Published:** 2022-09-26

**Authors:** Maha Abdallah Alnuwaiser

**Affiliations:** Department of Chemistry, College of Science, Princess Nourah Bint Abdulrahman University, P.O. Box 84428, Riyadh 11671, Saudi Arabia

## Abstract

Environmental pollution is one of the main factors that significantly affect biological systems and human health. Soil pollution with heavy metals is an increasingly pressing problem worldwide. In general, heavy metals are stable and do not decompose, unlike other organic pollutants. The quantity of them is natural components of soil crust, the remaining come from human activities, which may result from the extensive use of sewage. In the present study, a methodology aimed at simultaneous quantification of 16 heavy elements in soil of 3 different regions was developed. The concentration of 16 soil heavy metals (Se, Cd, V, Be, As, Mn, Co, Zn, Fe, Cr, Pb, Ni, Cu, Mo, Hg, and Ti) was measured in 11 sampling along Riyadh, Qassim, and Medina, Kingdom of Saudi Arabia from 3 sites soil treated with sewage water. These chemical minerals were identified in the samples using an ICPE-9000 spectrometer. The assessment of heavy metal contamination was derived using enrichment factors (EF), the pollution load index (PLI), and geoaccumulation index (*I*_geo_). This study revealed that the soil is predominantly polluted by Cd, As, and Mo of Riyadh and Medina and As, Mo, and Cd of Qassim region at site B and site C, respectively. As recorded, the highest concentration value of 5000 mg/kg for Fe at site (B) followed by Cu. The *I*_geo_ value of Cd is 1.1520 in Medina region. The *I*_geo_ value of Se is 3.2395 in Medina region, while its cumulative geographical index decreased in the regions of Riyadh and Qassim, which amounted to 2.6114 and 2.1699, respectively. The *I*_geo_ values of the rest of the minerals in the three regions studied indicated that the soil is unpolluted, while it was slightly to moderately polluted for both Mo and Hg in most regions studied. The minerals in the soil at all sites studied were less than the general average concentration. With the exception of mercury, molybdenum, arsenic, cadmium, and selenium, whose concentration exceeded the permissible and recommended limits. The increasing order of concentration of minerals was Be < V < Cd < Hg < Mo < Co < Zn < Pb < Cr < Se < As < Ni < Ti < Mn < Cu < Fe at all sites, respectively.

## 1. Introduction

Heavy metal toxicity is related with its accumulation in the soil. This leads to soil pollution. Soil pollution with heavy metals is an increasingly pressing problem worldwide, which may result from the extensive use of sewage for irrigation [1]. In general, heavy metals are stable and do not decompose unlike other organic pollutants [2]. Heavy elements are natural components of soil crust. However, human activities radically changed their geochemical and biochemical balance [3]. The increase of using toxic chemical compounds by people leads to an increase in the volume of wastewater [4]. Sewage water irrigation can contribute to the heavy metal amount in soil [5]. The food made from plants grown in sewage water is highly contaminated [6]. Wastewater contaminated with trace minerals, such as lead (Pb), zinc (Zn), copper (Cu), arsenic (As), chromium (Cr), molybdenum (Mo), boron (B), cobalt (Co), and manganese (Mn), many of them are unnecessary, but their buildup makes them toxic to plants, animals, and humans [7]. Using waste wastewater for a long time leads to an increase in the concentration of heavy metals in the soil [8, 9]. Soil consists of organic compounds and heterogeneous components of fluids and minerals that compose it [10]. The elements that man creates and leaves in the soil are greater than the elements from natural sources [11, 12].

Polluted water affects the soil. This effect is not only in industrial areas, but included even in agricultural fields, such as riverbeds [13–16]. Soil pollution and its toxicity are associated with high levels of heavy metals [17]. Concentrations of trace metals in sewage effluents vary from one city to another [18]. Despite the fact that the concentration of heavy metals in sewage effluents is low, the use of these wastewaters on agricultural lands for a long time results in the increase of levels of these metals in soils [18]. Contamination of toxic trace elements (TES) in agricultural soils is due to human activities [19]. Arsenic (As), lead (Pb), mercury (Hg), and cadmium (Cd), which are toxic, lead to some acute and chronic conditions [20]. Heavy metals are extremely hazardous to health as their accumulation in human and animal organisms causes severe hazards [21–24].

Remediation of these contaminated soils is due to human health and safe food production. Toxic metals minimized soil quality and affect plant productivity [25]. The presence of heavy metals in the soil leads to a significant change in its properties, which results in physiological, chemical, and biological changes in plants, which leads to reduced growth and thus reduces crop yield [26]. Irrigation with sewage water for a long time leads to changes in the soil due to the deposition of toxic elements [27]. There are a large number of reports [28, 29] showing the use of sewage water for irrigation is a major concern for the presence of toxic elements. Permanent irrigation with sewage water for agricultural lands led to food contamination [30].

Although wastewater contains small percentages of heavy elements (manganese, lead, iron, cadmium, and chromium), soil showed higher percentages due to the accumulation. Mineral accumulation in wastewater-irrigated soils in the following order: Fe > Mn > Pb > Cr > Cd [31]. The bioactivity of Cu, Zn, Ni, Cd, and Pd is significantly reduced in soils with a pH above 7 [32]. The industrialization of modern societies has created an exponential increase in the waste produced per person. In Saudi Arabia in 2016, solid waste are more than 6 million tons per year of solid waste in Riyadh, Jeddah, and Dammam [33]. UNESCO recognizes Jeddah as a historical city as a World Heritage Site [34, 35]. Environmental pollution is one of the obstacles when it comes to the revitalization and development of the city. Since 1962, Jeddah has been expanding rapidly. The largest pollution source is the sewage lake in Jeddah (east of Jeddah) since it contains toxic compounds due to water sedimentation in the residential area [36].

The objective of this work is to determine the soil contamination level of 16 heavy elements and compare them with the soil around the sewage plants and streams of Riyadh, Qassim, and Medina areas in the Kingdom of Saudi Arabia. These minerals were analyzed using the ICPE-9000 device.

## 2. Materials and Methods

### 2.1. Soil Materials

A total of 11 topsoil samples were collected from 3 different regions around the treated wastewater basin; region A represents the area on the wastewater basin; region B just 50 meters from the water basin of sewage plant; and region C just 100 meters from the sewage basin of Riyadh, Qassim, and Medina in Kingdom of Saudi Arabia. The soil was dried and sieved with a 2 mm sieve and left for a week at room temperature then placed in airtight plastic bags for preservation.

### 2.2. Methods

Various methods were applied to detect and evaluate heavy metals in the soil. Atomic Absorption (flame), Atomic Absorption (furnace), and Inductively Coupled Plasma (ICP) techniques were developed over the years for this purpose. Among the above methods, ICP is the more convenient method for qualitative and quantitative analysis. That is why this study had been designed to develop a high sensitivity, lower running cost, and the larger number of measured elements the more apparent time efficiency.

### 2.3. ICP Spectrometry Conditions

#### 2.3.1. ICP Spectrometry Parameters

Quantitative analysis was performed on a Shimadzu ICPE-9000 Spectrometer equipped with a highly efficient ionization and emission sources and CCD (charge-coupled device) detector. Its temperature was set at −14.89°C. Spectrum resolution, to avoid spectral interference was achieved automatically. A high-purity argon carrier gas was used. The flow rate of plasma gas (Ar) was maintained at 10 L/min, auxiliary gas (Ar) at 0.6 L/min, and carrier gas (Ar) at 0.7 L/min. The direction position AXIAL view, Rf power at 1.2 kW, pressure at 450 + 10 kPa. The rotation speed was adjusted to 20 rpm.

### 2.4. Preparation of Working Solution Standards

Working standard solutions were prepared by diluting a Scharlau ICP multi-element calibration standard solution in 5% HNO_3_ using deionized water to 1000 ml/L.

### 2.5. Preparation of Samples

To prepare soil samples wet digestion technique was performed by using concentrated acids. About 0.5 g of soil sample was taken into a clean and dry beaker. About 3 ml of conc. nitric acid and 1 ml of conc. hydrochloric acid were added to it. The resulting mixture was stored for 24 h. The mixture was placed in a heater at 150°C for 2 h. After cooling to room temperature, the mixture was filtered into a 500 ml volumetric flask, its volume adjusted up to the mark with deionized water.

### 2.6. Analysis of Heavy Metals of Soil Samples

#### 2.6.1. Physical and Chemical Properties of the Soil Sample

The acidity and soil contamination level of the proposed method was determined by measuring the mineral concentration (pH), metal concentration in terms of mg/kg, the conductivity (EC) in terms of *μ*s/cm, values of total dissolved solids (TDS) in terms of *µ*g/L, and chlorine anion (Cl^−^) concentration in terms of *µ*g/L.

### 2.7. Statistical Analyses

To find out the significance and significant differences of soil sample data, statistical analysis was performed by means of a test ANOVA.

#### 2.7.1. Contamination Assessment Methods

To assess soil enrichment and pollution caused by minerals, Pollution Load Index (PLI) enrichment factors (EF) in addition to the geoaccumulation index (*I*_geo_) were used.

*(1) Assessment of Heavy Metal Pollution.* To assess the contamination degree and pollution of the proposed method, concentration levels of samples [37] were determined using (PLI) pollution load index. The pollution load index is measured by comparing the concentration value of the sample to the value of the mineral background in the soil. The PLI was determined [37] as follows:

(1) $$\begin{array}{c} \text{PLI}={\left(P_{i_{1}}\times P_{i_{2}}\times P_{i_{3}}\times \ldots \times P_{i_{n}}\right)}^{1/n}, \end{array}$$

where PLI is the contamination level; *P*_*i*_ is the stand for single element contamination index *i*; and *n* is the number of elements.

(2) $$\begin{array}{c} P_{i}=\frac{C_{i}}{S_{i}}, \end{array}$$

where *P*_*i*_ is the stand for single element contamination index *i*; *C*_*i*_ is the concentration of the element in the sample; and *S*_*i*_ is the posterior focus of the sample.The value PLI > 1 indicates a contaminated site; the value of PLI < 1 indicates a contaminated site in the absence of pollution.

#### 2.7.2. Quantitative Measurement of Mineral Pollution

To measure the extent of metal contamination by the proposed method, geoaccumulation Index (*I*_geo_) was determined by comparing the concentration of the metal sample in the soil with the geographical accumulation parameter. *I*_geo_ has been calculated [38] as follows:

(3) $$\begin{array}{c} I_{\text{geo}}=\;\log_{2}\left(\frac{C_{n}}{1.5B_{n}}\right), \end{array}$$

where *C*_*n*_ is the measured total concentration of the element *n* in the soil; *B*_*n*_ is the average concentration of element *n* geochemical background parameter; and 1.5 is the constant used to reduce the effects of potential changes in soil background values.*I*_geo_ ≤ 0 indicates unpolluted; 0 < *I*_geo_ < 1 indicating unpolluted/moderately polluted; 1 < *I*_geo_ < 2 moderately polluted; 2 < *I*_geo_ < 3 indicating moderately/strongly polluted; 3 <*I*_geo_ < 5 indicating strongly polluted; 4 < *I*_geo_ < 5 indicating strongly/extremely polluted; and *I*_geo_ > 5 indicating extremely polluted [38].

#### 2.7.3. Assessment of Soil Enrichment

To assess the presence and intensity of anthropogenic contaminant deposition on surface soil enrichment factor (EF) as an indicator was calculated by normalization of iron [39–42] concentration in the topsoil with respect to the concentration of a reference element. EF is calculated [43] as follows:

(4) $$\begin{array}{c} \text{EF}=\frac{{\left(C_{x}/C_{\text{reference}}\right)}_{\text{sample}}}{{\left(C_{x}/C_{\text{reference}}\right)}_{\text{background}}}, \end{array}$$

where EF is the enrichment factor; *C*_*x*_ is the concentration of the element of interest; and *C*_Fe_ is the concentration of a reference element (Fe) for the purpose of normalization.

EF < 2 represents a minimal deficiency of the element, moderate: 2 < EF < 5, significant: 5 < EF < 20, strong: 20 < EF < 40, and extremely high enrichment: EF < 40.

## 3. Results and Discussion

### 3.1. Analysis of Heavy Metals of Soil Samples

#### 3.1.1. Physical and Chemical Properties of the Soil Sample

The pH and electrical conductivity values of soil as shown in Table 1 are ranged between 5.8 to 7 and 1.02 to 41.2 *μ*s/cm, 6.4 to 7.3 and 6.7 to 2.51 *μ*s/cm, and 6.8 to 7.5 and 0.39 to 2.6 *μ*s/cm at stream site A (represents the position at the edge of the sewage stream), B (represents the right of the edge (outside the sewage stream) at a distance of 50 m), and C (at the right of the edge (outside the sewage stream) at a distance of 100 m), respectively. pH values are within the allowable limit [44, 45], except at site A of Qassim region (5.8). On variation with distance away from sewage stream, the highest soil pH level with continuous irrigation with sewage water can cause an increase in sulfate levels in wastewater [46, 47]. The electrical conductivity of soil contaminated with sewage water in most of the samples exceeded the value of 1 *μ*s/cm, which indicates that this soil is salty in nature. The total dissolved solids (TDS) values at three sites as shown in Table 1 varied greatly. The highest (TDS) values are 7165 and 11845 mg/L observed at site A of Qassim and Medina, respectively, while that far from sites B and C are significantly decreased. The highest Cl^−^ anion concentration (1189.9 mg/L) was observed at sewage stream of Qassim region. Generally decreasing soil pH was observed, it could be due to higher inputs of organic matter as the result of sewage irrigation [48]. The results shown in Table 1 indicate that the mobility of heavy metals decreases with increasing soil pH it could be due to the precipitation of hydroxides or carbonates from insoluble organic complexes.

### 3.2. ICP Spectrometry Parameters

#### 3.2.1. Analysis of Heavy Metals of Soil Samples

*(1) Metals at Sewage Soil of Riyadh.* The concentration of Cd, V, Be, Co, Zn, Cr, Pb, Mo, and Hg in the soil shown in Table 2 ranges from 0.1 to 2.05 mg/kg at Riyadh regions around the sewage site (A, B, and C), which indicate that its concentrations are lower than other minerals. While the concentration of Se, As, Mn, Ni, and Ti increased, are ranged between 3.4 and 5.5 mg/kg. The concentration of Cu is 10 mg/kg, which indicates a high concentration, while the concentration of Fe is 445 mg/kg at this site, which indicates the highest mineral concentration. The concentration of all minerals in the soil is less than the global average concentration at sewage stream site A, while that of Se, Cd, and Hg are 18, 4, and 13 times higher, respectively. The results are shown that there was a discrepancy in the concentration of minerals in the soil at a distance of 50 m away from the sewage stream (region B).

In general, the increasing order of concentrations of minerals was Fe > As > Cu > Mn > Se > Ti > Ni > Zn > Co > Mo > Pb > Cr > Hg > Cd > V > Be and within the permissible limit in the soil except that of Se, Cd, As, Mo, and Hg. Their proportions in the soil were higher than the soil recommended limit of 100 m from the sewage stream site C. The concentration of Fe is 750 mg/kg at site C, which indicates a high concentration, followed by Cu with a concentration of 9 mg/kg, Mn and Se have the same concentration of 6.5 mg/kg. The concentrations of other elements ranged between 0.165 and 4.8 mg/kg. All the elements are within the range of the global average of minerals in the soil except mercury, cadmium, and selenium, where their concentrations are 16, 4, and 21 times higher than the permissible limit in the soil, and molybdenum exceeded the permissible limit in this site with a slight increase. On making a comparison of concentrations of minerals in the three sites (A, B, and C) in this area the concentrations of minerals at site B, are the highest for all minerals except that of selenium, the highest concentration of selenium observed at the site C. The results show that the mineral content at site C is higher than that at site A. The decreasing order of observing minerals at sites was A < C < B. The highest concentrations of minerals at the three sites are iron, copper, arsenic, and manganese, respectively. The concentration of arsenic in the soil at site B is higher than that at sites A and C, which indicate that the safe limit is exceeded in the soil at the site B. The concentration of molybdenum also exceeded the recommended limit in the soil at the sites C and B only. The concentrations of mercury, cadmium, and selenium exceeded the permissible concentration limit in the soil at three sites, while the concentrations of the rest of the minerals are within the allowed permissible limit.

### 3.3. Metals at Sewage Soil of Qassim

The concentration of the mineral in the soil at sites A, B, and C of Qassim region is shown in Table 2. The concentration of Fe in the soil is 550 mg/kg at sewage site A, which indicates the highest one, followed by Cu; the lower one is that of Mg at ranged from 8.5 to 7 mg/kg. The decreasing order of concentrations of minerals was Ti > Se > Ni > As > Pb > Mo > Cr > Zn > Co > Hg > Cd > Be > and V. The concentrations of all minerals in the soil within the allowed limit except that of Hg, Cd, and Se, which are 12, 4, and 16, times higher than the global average of metal concentration [49], respectively. The concentrations of Cd, V, Pb, Be, Co, Zn, Cr, Ni, Hg, and Mo in the soil are ranged from 0.13 to 2.7 ppm at site B, which indicate low concentration, while that of Ti and Se are increased which are 4.6 and 4.05 ppm, respectively. The concentrations of Cd, V, Cr, Be, Co, Zn, Pb, Ni, Mo, and Hg in the soil ranged from 0.13 to 2.7 mg/kg at site B. The concentrations of Mn, As, and Fe in the soil at site B are 5.5, 5.5, and 420 ppm, respectively. The concentrations of all minerals at site B are within the allowed limit except that of mercury, arsenic, cadmium, and selenium, which have higher levels than the global average value of minerals in the soil. The mineral amount in the soil varied with respect to the site C. The concentrations of Fe and Mn in the soil at site C are 1900 and 30.5 ppm, respectively, while the concentrations of other minerals studied at site C ranged from 0.18 to 6 ppm. The concentrations of all minerals in the soil at site C are within the safe allowed limit in the soil except that of mercury, cadmium, and selenium are 13, 10, and 20 times higher than the global average value of minerals in the soil, respectively. Molybdenum and arsenic exceeded the recommended limit in soil when comparing the mineral content of three sites (A, B, and C).

The results shown in Table 2 indicate that the concentrations of all minerals in the soil at site C are significantly highest. The increasing order of minerals content in Qassim region is B < A < C. The high concentration of metals at site C could be due to human factors and the influence of winds in this region. Iron metal represents the highest concentration of minerals at the three sites (A, B, and C) and a significant increase in manganese concentration was observed at site C which is 30.5 mg/kg as compared to its concentration at sites B and A which are 7 and 5.5 ppm, respectively. The concentration of Copper is high at the three sites, and moderate concentrations of arsenic and selenium are observed. The concentrations of all minerals were less than the permissible values in the soil except for mercury, cadmium, and selenium whose concentration exceeded the recommended limit in the soil of the three sites (A, B, and C), while arsenic exceeded the permissible concentration at the two sites (C and B). Only, the molybdenum concentration exceeded the permissible safe limit in the soil at site C.

### 3.4. Metals at Sewage Soil of Medina

The mineral content of Medina region in the soil at sites (A, B, and C) is shown in Table 2, indicating that the concentrations of mineral in the soil at three sites are different. The concentrations of Ti, Fe, Cu, and Mn in the soil at site A are 1300, 19.5, 16.5, and 11 mg/kg, respectively, which indicate high concentrations. The concentrations of Ni and As at site A are 5.5 and 4.7 mg/kg, respectively, which indicate moderate concentration, while the concentrations of the other metal studied at site A ranged between 0.165 and 3 mg/kg. The concentrations of all minerals in the soil are less than the corresponding value in the soil [49], except that of Se, Cd, and Hg, which are 14, 6, and 18 times higher than the permissible concentration in the soil recommended limit, respectively, while other minerals are within the safe limit in the soil. Very high concentrations of Fe, Mn, Cu, and Ti are 5000, 100, 28, and 19 mg/kg, respectively, in the soil observed at site B. A moderate concentration ranging between 0.165 and 3 mg/L was observed at site B. By comparing the concentrations of minerals in the soil at site C, the results showed a large difference in the concentrations of minerals in the soils due to the large disparity in the concentration of Fe, Mn, Ti, and Cu which are 4350, 70, 28, and 21 mg/kg, respectively, compared with the concentration of Hg, Be, V, and Cd which are 0.485, 0.24, 0.7, and 0.9 mg/kg, which indicate that the concentrations in the soil are within the safe and permissible limit (<1 mg/kg) except that of Hg, Mo, Cd, and Ce which have highest concentration 16, 2, 15, and 27 times higher than the order of limit in the soil. The results shown in Table 2 and Figure 1 indicate that the concentrations of all minerals in three cities at site B are the highest, except that of titanium, with the highest concentration of it (28 mg/kg) observed at site C. The decreasing order of minerals content in Medina region is B < A < C.

The results of the study indicated that iron, manganese, titanium, and copper are the most abundant minerals in the three areas. The concentration of manganese in the soil at site A is 16.5 mg/kg and in the soil at site is 100 mg/kg. Moderate concentrations of minerals in the soil at the three sites are nickel, chromium, zinc, arsenic, and silicon, while the rest of the minerals have lower concentrations (in the range between 0.25 and 5.5 mg/kg). The concentration of mercury, molybdenum, cadmium, and selenium exceeded the global average concentration, while the concentration of other metals remain within the permissible limit, which indicated safety in the soil.

### 3.5. Comparison of Mineral Concentrations at Different Sites

The results shown in Table 3 indicate that differences in mineral concentration depend on their location at the stream of the sewage. The highest concentration of all minerals was observed in the soil at site B of Riyadh and Medina and site C of Qassim. The highest concentration was observed in Fe (5000 mg/kg) at site B of Medina, the lowest value is 420 mg/kg at site B of Qassim, indicating the prevalence of iron metal in three regions studied. Iron having a high concentration irritates the digestive system and changes the taste of water by promoting iron bacteria [50]. A similar trend was observed in Cu (as an essential nutrient) in the soil close to the sewage stream, indicating contaminated soil. The exposure to copper concentrations for long periods causes liver and kidney and anemia diseases [51]. The third mineral abundant was observed in Mn at site B of Medina and site C of Qassim. Eating Manganese has a daily need in a small amount that is important to maintain good health [52]. A high concentration was observed in Ti at the three sites in Medina region and at three sites of Riyadh and Qassim. The concentration of Cr is ranging between 1.75 and 5.5 mg/kg at all sites of three regions, chromium is considered a toxic metal to all living organisms. The level of toxic chromium in the soil is 50 parts per million [53]. The concentration of Ni at all sites ranged between 2.7 and 10.5 mg/kg. Nickel is considered a human carcinogen when ingested in higher than normal concentrations. Nickel is the main cause of allergic contact dermatitis, especially for women [54].

Human inputs such as manure and fertilizers contain lower levels of nickel and chromium than those already in the soil [55]. The concentration of Zn ranged between 0.75 and 4.8 mg/kg at all sites. Zinc is an essential element, but high levels of it can cause adverse health effects. The concentration of Co and Pb is low and moderate, respectively, and the least concentration of Be and V were observed at all sites studied. The minerals in all the locations of the studied areas were less than the general average concentration according to Lindsay 1979 with the exception of mercury metal, whose concentration is within the range 0.365 to 0.55 mg/kg, exceeded the permissible limit in all regions. The level of molybdenum also exceeded the permissible limit in all sites, whose concentration ranged between 2.3 and 4.3 mg/kg, except at sites B and A of Qassim region and site A of Riyadh region. Molybdenum is an essential element in animal and plant nutrition [56]. The concentration of As exceeded the permissible limit in the soil at all sites except at site A of Medina region, at site A of Qassim region, and at site C of Riyadh region. Arsenic is the main constituent of some pesticides and fertilizer substances of soil [57].

The concentration of Cd is higher than the permissible and recommended limit in the soil at sites. The highest value is 8.5 mg/kg in the soil at site B of Medina region, the lowest concentration is 4.8 mg/kg was observed at site A of Qassim region. Cadmium is a highly toxic metal, that cause many symptoms such as nausea, vomiting, difficulty breathing, convulsions, and loss of consciousness. Chronic exposure to high doses of cadmium causes anemia, cardiovascular disease, kidney problems, and high blood pressure [58]. The concentration of Se (4.05–8.5 mg/kg) exceeded the limit at all sites studied. The increase in selenium concentration may be due to the addition of selenium to fertilizers. Precipitation also plays a key role in determining the surface soil level content [59]. In general, the increasing order of concentration of minerals was Be < V < Cd < Hg < Mo < Co < Zn < Pb < Cr < Se < As < Ni < Ti < Mn < Cu < Fe at all sites, respectively.

### 3.6. Statistical Analysis

Table 3 is a summary of the minimum, maximum, average, and standard deviation of the number of metal ions in soil samples collected from sanitation sites for three regions of the Kingdom of Saudi Arabia. By looking at the results of Table 3, we find the discrepancy in the range of all distributions of minerals compared with their means, respectively. It is an indication of the contamination of the sample with these minerals studied except for cadmium, arsenic, selenium, molybdenum, and mercury. The decreasing trend of averages of metal levels was as follows: As > Se > Hg > Mo > Cd mg/kg concentrations [59, 60].

### 3.7. Contamination Assessment Methods

#### 3.7.1. Assessment of Soil Enrichment

Table 4 is a summary of the minimum, maximum, mean, and standard deviation for heavy items in 30 soil samples collected at treated wastewater basin soil of Riyadh, Medina, and Qassim, Kingdom of Saudi Arabia. The enrichment factors (EF) of Cr, Ti, V, Mn, and Zn concentration in the soil as shown in Table 4 ranged from 0.06 to 1.91 (EF < 2) in three regions studied, which indicates that the soil is uncontaminated by these elements, and metals are entirely to crustaceans and natural processes. The enrichment factors (EF) of Be and Ni concentration ranged from 2 to 5 (2 < EF < 5) at site of Riyadh and Qassim, which shows moderate fertilization, while their enrichment in the soil of Medina reached the minimum level of the presence of the element. The behavior of Cu shows that the enrichment factors (EF) ranged from 5 to 20 at the sites of Riyadh and Medina, which indicates significant fertilization, while it was fertilized strongly in Qassim region. The enrichment factors (EF) of Cd, As, and Mo concentrations of Riyadh and Medina indicate strong fertilization, while high value of EF (EF > 40) of Qassim region indicates the possibility of severe extreme pollution for As, Mo, and Cd. A relatively higher value of EF (EF > 40) of Se concentrations in three regions studied, leads to severe soil contamination of this element. The difference in the EF values in the analyzed soil samples reflects anthropogenic effects, which might be a difference in the input volume of each mineral in the soil. Enrichment factors (EF) values of heavy metals in soil samples collected at treated wastewater basin soil of Riyadh, Medina, and Qassim are shown in Figure 2.

### 3.8. Assessment of Heavy Metal Pollution

The results of Pollution Index (PI) values of heavy elements of Riyadh, Qassim, and Medina are shown in Table 5 and Figures 3 and 4. Table 5 is a summary of the low, high, and mean values of all heavy values elements found in the soil at site B of Riyadh, Qassim, and Medina regions. The Pollution Index (PI) values of Ti, Cu, Ni, Pb, Cr, Zn, Co, Mn, Be, and V ranged from 0.0010 to 0.9000 (PI < 1) with an average range between 0.0012 and 0.3704, which indicate that the soil is unpolluted. The PI value of Hg, Mo, and As of Riyadh and Medina ranged from 1.0000 to 1.6538 (PI > 1) with an average range between 0.8205 and 1.1375 which indicate that the soil is slightly polluted in these two regions, while the PI values of these elements of Qassim are PI < 1 which indicate that the soil is unpolluted. The value of As of Medina is 3.3333 (PI > 1) which indicate that the soil is strongly polluted, while its presence in the soil of the regions of Riyadh and Qassim is considered unpolluted. The PI value of Se is ranged from 6.7500 to 14.1667 (PI > 1) with an average of 10.0278, which indicate that the soil is very strongly polluted.

### 3.9. Quantitative Measurement of Mineral Pollution

Quantitative measurement of mineral pollution of the soil studied is shown in Table 6 and Figure 5. The geographical accumulation index (*I*_geo_) value of Mo is 0.1409 (*I*_geo_ < 0) of Riyadh and Qassim, which indicate that the soil is unpolluted. The *I*_geo_ value of Cd is 1.1520 (*I*_geo_ > 1) of Medina region which indicate that the soil is moderately polluted, while it did not give pollution in the regions of Riyadh and Qassim. Cd is considered one of the most dangerous toxic minerals and accumulates significantly in soil samples. The *I*_geo_ value of Se is 3.2395 (*I*_geo_ > 1) of Medina region which indicate that the soil is strongly polluted, while its cumulative geographical index decreased in the regions of Riyadh and Qassim, which amounted to 2.6114 and 2.1699, respectively, that classified the pollution of this mineral in these two regions as moderately to highly polluted. The *I*_geo_ values of the rest of the minerals in the three regions studied are indicated that the soil is unpolluted as shown in Figure 5. The calculated values refer to the (PI) pollution index and geographic cumulative index (*I*_geo_) from medium to high pollution levels from Se in the soil of all regions studied. It was also found that this soil was polluted with As of Medina region. While it was slightly to moderately polluted for both Mo and Hg in most regions studied.

## 4. Conclusion

A sensitive, reproducible, and relatively simple ICP method was developed to screen and quantify heavy metals that cause soil pollution. Samples collected from regions without any information about levels of contamination of the soil. From the collected samples, around 31% of samples (mercury, molybdenum, arsenic, cadmium, and selenium) found whose concentration exceeded the permissible and recommended limits. This finding demonstrated the importance of soil constituents in fertilization and cultivation processes.

## Figures and Tables

**Figure 1:** The average concentration (mg/kg) of heavy metals at sites A, B, and C of Riyadh, Qassim, and Medina.

**Figure 2:** EF value for heavy metals in soil samples collected from Riyadh, Qassim, and Medina regions.

**Figure 3:** Variations of PI value in the soil samples from Riyadh, Qassim, and Medina.

**Figure 4:** The percentage of PI in each metal in the study area.

**Figure 5:** The value of *I*_geo_ for each metal in soil of Riyadh, Medina, and Qassim.

**Table 1:** Results of physical and chemical properties of soil study for areas (A, B, and C) in the cities of Riyadh, Qassim, and Medina.

Region		pH	EC (ms/cm)	TDS (*μ*g/L)	Cl^−^ (*μ*g/L)
Riyadh	Area (A) soil	7.0	1.02	275	45.67
	Area (B) soil	6.7	2.51	680	112.92
	Area (C) soil	6.8	2.6	705	117.08

Qassim	Area (A) soil	5.8	26.4	7165	1189.9
	Area (B) soil	7.3	0.67	180	29.89
	Area (C) soil	7.5	0.39	105	17.43

Medina	Area (A) soil	6.8	41.2	1845	306.4
	Area (B) soil	6.4	2.05	555	92.16
	Area (C) soil	6.9	1.60	435	72.24

**Table 2:** Results of heavy element concentration (mg/kg) at sites A, B, and C of Riyadh, Qassim, and Medina regions.

Element	Riyadh			Qassim			Medina		
	Area (A)	Area (B)	Area (C)	Area (A)	Area (B)	Area (C)	Area (A)	Area (B)	Area (C)
Ti	3.4	5.5	4.75	5.5	4.6	12	19.5	19	28
Hg	0.39	0.475	0.485	0.365	0.34	0.41	0.415	0.55	0.485
Mo	1.85	2.6	2.3	1.9	1.8	3.55	2.7	4.3	4.15
Cu	10	13	9	8.5	8.5	13.5	11	28.5	21
Ni	4	5	4.8	4.25	2.7	8	5.5	10.5	9
Pb	2	2.55	2.55	2.05	1.95	3.7	3	5.5	4.75
Cr	2.05	2.5	1.95	1.75	1.45	3.3	2.25	7	5.5
Fe	445	1250	750	550	420	1900	1300	5000	4350
Zn	1.95	4.8	1.15	1.15	0.75	2.75	1.8	9	6
Co	0.75	4.65	1.15	0.9	0.65	2.85	2.25	5.5	3.8
Mn	3.85	11.5	6.5	7	5.5	30.5	16.5	100	70
As	4.55	13.5	4.65	3.6	5.5	7.5	4.7	13	7
Be	0.135	0.16	0.165	0.145	0.145	0.18	0.165	0.305	0.24
V	0.1	0.21	0.175	0.11	0.13	0.37	0.25	1	0.7
Cd	0.225	0.27	0.24	0.255	0.205	0.6	0.36	1	0.9
Se	5.5	5.5	6.5	4.8	4.05	6	5.5	8.5	8

**Table 3:** Results of the soil contaminated with heavy metals at wastewater of Riyadh, Qassim, and Medina regions.

Element	Min	Zone	Max	Zone	Mean	SD	SE
Ti	4.6	Qassim	19	Medina	9.7000	8.0666	4.6573
Hg	0.34	Qassim	0.55	Medina	0.4550	0.1064	0.0614
Mo	1.8	Qassim	4.3	Medina	2.9000	1.2767	0.7371
Cu	8.5	Qassim	28.5	Medina	16.6667	10.4921	6.0576
Ni	2.7	Qassim	10.5	Medina	6.0667	4.0079	2.3140
Pb	1.95	Qassim	5.5	Medina	3.3333	1.9002	1.0971
Cr	1.45	Qassim	7	Medina	3.6500	2.9483	1.7022
Zn	0.75	Qassim	9	Medina	4.8500	4.1252	2.3817
Co	0.65	Qassim	5.5	Medina	3.6000	2.5899	1.4953
Mn	5.5	Riyadh	100	Medina	39.0000	52.9127	30.5491
As	5.5	Qassim	13.5	Riyadh	10.6667	4.4814	2.5874
Be	0.145	Qassim	0.305	Medina	0.2033	0.0884	0.0510
V	0.13	Qassim	1	Medina	0.4467	0.4809	0.2776
Cd	0.205	Qassim	1	Medina	0.4917	0.4414	0.2549
Se	4.05	Qassim	8.5	Medina	6.0167	2.2695	1.3103

**Table 4:** Results of enrichment factor at soil of Riyadh, Qassim, and Medina regions treated with sewage water.

Element	Min	Zone	Max		Mean	SD	Pollution level
Ti	0.0390	Medina	0.1124	Qassim	0.0655	0.0407	Light
Hg	12.9800	Medina	95.5238	Qassim	51.1146	41.6281	Extreme
Mo	15.6123	Medina	77.8022	Qassim	43.7248	31.5211	Extreme
Cu	5.9787	Medina	21.2275	Qassim	12.7049	7.7815	Significant
Ni	1.4576	Medina	4.4622	Qassim	2.8988	1.5060	Moderate
Pb	2.5960	Medina	10.9571	Qassim	6.1225	4.3313	Significant
Cr	0.7342	Medina	1.8106	Qassim	1.1979	0.5534	Light
Zn	0.8872	Qassim	1.9079	Riyadh	1.2298	0.5872	Light
Co	2.7326	Medina	9.2413	Riyadh	5.2728	3.4814	Significant
Mn	0.5109	Riyadh	1.1106	Medina	0.7829	0.3037	Light
As	9.4400	Medina	47.5458	Qassim	32.0660	20.0328	Strong
Be	0.9597	Medina	5.4317	Qassim	2.8018	2.3378	Moderate
V	0.0610	Riyadh	0.1124	Qassim	0.0820	0.0269	Light
Cd	31.4667	Qassim	76.7937	Qassim	47.4148	25.4740	Extreme
Se	6.1723	Qassim	35.0110	Qassim	412.8127	317.7110	Extreme

**Table 5:** Results of pollution indexes of Riyadh, Qassim, and Medina regions soil treated with sewage water.

Element	Min	Zone	Max	Zone	Mean	SD	Classification range of pollution level
Ti	0.0010	Qassim	0.0041	Medina	0.0021	0.0018	Unpolluted
Hg	0.8500	Qassim	1.3750	Medina	1.1375	0.2660	Slightly polluted
Mo	0.6923	Qassim	1.6538	Medina	1.1154	0.4910	Slightly polluted
Cu	0.1889	Qassim	0.6333	Medina	0.3704	0.2332	Unpolluted
Ni	0.0397	Qassim	0.1544	Medina	0.0892	0.0589	Unpolluted
Pb	0.0975	Qassim	0.2750	Medina	0.1667	0.0950	Unpolluted
Cr	0.0161	Qassim	0.0778	Medina	0.0406	0.0328	Unpolluted
Zn	0.0079	Qassim	0.0947	Medina	0.0511	0.0434	Unpolluted
Co	0.0342	Qassim	0.2895	Medina	0.1895	0.1363	Unpolluted
Mn	0.0065	Qassim	0.1176	Medina	0.0459	0.0623	Unpolluted
As	0.4231	Qassim	1.0385	Medina	0.8205	0.3447	Unpolluted
Be	0.0483	Qassim	0.1017	Medina	0.0678	0.0295	Unpolluted
V	0.0010	Qassim	0.0077	Medina	0.0034	0.0037	Unpolluted
Cd	0.6833	Qassim	3.3333	Medina	1.6389	1.4714	Slightly polluted
Se	6.7500	Qassim	14.1667	Medina	10.0278	3.7826	Very strongly polluted

**Table 6:** Results of geographical accumulation index (*I*_geo_) of Riyadh, Qassim, and Medina regions. Soil treated with sewage water.

Element	Min.	Zone	Max.	Zone	Mean	SD	Classification range of pollution level
Ti	−0.5507	Qassim	−8.50445	Medina	−0.7827	1.1145	Unpolluted
Hg	−0.8194	Qassim	−0.12553	Medina	−0.4273	0.3557	Unpolluted
Mo	−1.1155	Qassim	0.140862	Medina	−0.5199	0.6307	Unpolluted
Cu	−2.9894	Qassim	−1.244	Medina	−2.2032	0.8855	Unpolluted
Ni	−5.2395	Qassim	−3.280107	Medina	−4.2900	0.9811	Unpolluted
Pb	−3.9434	Qassim	−2.44745	Medina	−3.3158	0.7765	Unpolluted
Cr	−6.5408	Qassim	−4.269460	Medina	−5.5217	1.1535	Unpolluted
Zn	−7.5699	Qassim	−3.984893	Medina	−5.4822	1.8640	Unpolluted
Co	−5.4544	Qassim	−2.37345	Medina	−3.4812	1.7131	Unpolluted
Mn	−7.8569	Qassim	−3.672425334	Medina	−6.1073	2.1748	Unpolluted
As	−1.8260	Qassim	−0.530514717	Riyadh	−0.9805	0.7327	Unpolluted
Be	−4.9558	Qassim	−3.883043849	Medina	−4.5509	0.5827	Unpolluted
V	−0.5507	Qassim	−7.60733035	Medina	−9.3390	1.5390	Unpolluted
Cd	−1.1343	Qassim	1.152003093	Medina	−0.2398	1.2216	Unpolluted
Se	2.1699	Qassim	3.2395	Medina	2.6736	0.5375	Moderately-strongly polluted

## Data Availability

The data used to support the findings of this study are included within the article. The used materials are available in the Princess Nourah bint Abdulrahman University store.
